# LINC00978 promotes hepatocellular carcinoma carcinogenesis partly via activating the MAPK/ERK pathway

**DOI:** 10.1042/BSR20192790

**Published:** 2020-03-09

**Authors:** Quan Zhang, Shujie Cheng, Liye Cao, Jihong Yang, Yu Wang, Yaqing Chen

**Affiliations:** 1 Department of Surgery, The Affiliated Hospital of Hebei University, Baoding, Hebei 071000, P.R. China; 2 Hebei University School of Medicine, Baoding, Hebei 071000, P.R. China

**Keywords:** carcinogenesis, hepatocellular carcinoma, LINC00978, Long non-coding RNA, MAPK/ERK pathway

## Abstract

**Objective**: To study the role of long non-coding RNA (lncRNA) LINC00978 in hepatocellular carcinoma (HCC) carcinogenesis.

**Materials and methods**: LINC00978 expression level was measured by reverse transcription quantitative real-time PCR (RT-qPCR) in HCC tissues and adjacent healthy liver tissues from 49 HCC patients. MTT assay, colony forming assay, and flow cytometry were performed to evaluate the effects of shRNA-mediated LINC00978 knockdown on HCC cell proliferation, cell cycle progression, and apoptosis *in vitro*. Xenograft tumor model was performed to determine the effects of LINC00978 knockdown on HCC tumor growth *in vivo*. Western blot was used to assess the activation of signaling molecules in the apoptosis and mitogen-activated protein kinase (MAPK)/extracellular signal-regulated kinase (ERK) pathway.

**Results**: LINC00978 expression was significantly up-regulated in human HCC tissue relative to adjacent normal tissue, and LINC00978 high expression was correlated with poor HCC overall survival. LINC00978 was up-regulated in HCC cell lines. ShRNA-mediated LINC00978 knockdown significantly decreased HCC cell proliferation, and induced HCC cell cycle arrest and apoptosis *in vitro*. LINC00978 knockdown led to significant decrease in tumor xenograft size *in vivo*. Western blots revealed LINC00978 inhibition decreased ERK, p38, and c-Jun N-terminal kinase (JNK) phosphorylation in HCC cells.

**Conclusions**: LINC00978 is highly expressed in human HCC tissue and correlates with poor HCC prognosis. LINC00978 promotes HCC cell proliferation, cell cycle progression, and survival, partially by activating the MAPK/ERK pathway. Our findings partially elucidated the roles of LINC00978 in HCC carcinogenesis, and identified a therapeutic target for HCC.

## Introduction

Hepatocellular carcinoma (HCC) is the most common primary malignancy of the liver, and the most common cause of death in people with chronic liver disease and cirrhosis [1]. In contrast with the overall decline for most major cancers, the death rates of HCC rose by 1.6–2.7% per year from 2011 to 2015 for both women and men [2], and it is expected to continue to rise in the coming years [3]. Currently, HCC is the second leading cause of cancer deaths worldwide [4,5]. In China, 466100 HCC cases are newly diagnosed each year, accounting for over 50% of global incidences [6,7]. The incidence of HCC is higher in Asia and Africa comparing with other regions, which is largely due to the high prevalence of hepatitis B infection and exposure to aflatoxin. More recently, there have been steady increases in HCC in the developed countries due to an increase in hepatitis C infection [2]. Current treatment for HCC is limited to surgical resection and liver transplantation, with no effective systemic therapies. The overall outcome is poor, with more than 50% of patients suffering from recurrence and metastasis, as well as death within 3–6 months. Therefore developing novel, efficacious diagnostic and therapeutic strategies for HCC becomes a major public health demand.

Long non-coding RNAs (lncRNAs) participated in carcinogenesis, and offered valuable information in early diagnosis and prognosis [8–10]. lncRNAs are a diverse class of non-protein-coding RNA molecules with over 200 nucleotides in length. The human transcriptome is enriched for lncRNAs, containing nearly 30000 different transcripts that far outnumber protein coding transcripts [10]. LncRNAs can be classified into five subtypes based upon their genomic organization: intergenic, intronic, antisense, bidirectional, and enhancer lncRNAs [10]. Several mechanisms that govern how lncRNAs regulate cellular functions have been described [11,12], including directly affecting the chromatin architecture, or binding to regulatory RNAs or proteins. The aberrant expression of several lncRNAs have been identified in HCC, including HOTAIR [13,14], MALAT1 [15], HULC [16,17], XIST [18], MEG3 [19], HEIH [20,21], and PANDA [22], some of which have displayed potential values in prognosis or a causal role in tumorigenesis [10]. However, to date, the vast majority of HCC-relevant lncRNAs have not been characterized in detail.

Recently, LINC00978 (also known as MIR4435-2HG, AGD2, or MORRBID) was identified as a novel lncRNA that promotes lung cancer growth [23] and acts as a biomarker for gastric [24] and breast cancer patients [25]. LINC00978 transcription was correlated with stem cell differentiation [26], and its murine ortholog, *Morrbid*, promotes myeloid cell lifespan [27], suggesting a pro-survival role for this lncRNA. However, the functional significance of LINC00978 in HCC has never been studied.

Here we showed that LINC00978 plays a critical role in HCC carcinogenesis *in vitro* and *in vivo*. LINC00978 expression was up-regulated in HCC tissue compared with normal liver tissue, and it was associated with poor HCC prognosis. LINC00978 promoted HCC cell proliferation, inhibited apoptosis *in vitro*, and enhanced tumor growth *in vivo*, partially by activating the mitogen-activated protein kinase (MAPK)/extracellular signal-regulated kinase (ERK) pathway. Our study suggests that LINC00978 may be an oncogene in HCC, and could offer potential prognostic value for HCC patients.

## Materials and methods

### Patients and samples

Liver tumor tissue and matched adjacent healthy liver tissues were from 49 HCC patients that underwent surgeries at Hebei University between February 2010 and July 2011. All tissues were snap-frozen in liquid nitrogen immediately following excision during the surgery and stored at −80°C until analysis. Two pathologists confirmed pathological diagnosis of all exercised tissues. Clinicopathological parameters of all recruited HCC patients were documented. The protocols were approved by the Ethics Committee of the Hebei University. Written informed consent was obtained from all patients from whom tissue samples were collected.

### Cell lines and culture

Normal human hepatic cell line LO2 and human HCC cell lines SK-Hep1, Bel-7404, Huh7, Hep3B, and HepG2 were obtained from the American Type Culture Collection (ATCC, U.S.A.). LO2 cell was cultured in DMEM medium (Gibco, U.S.A.) containing 10% fetal bovine serum (FBS; Hyclone, U.S.A.), 100 U/ml penicillin and 100 μg/ml streptomycin. HCC cell lines were cultured in RPMI-1640 medium (Gibco, U.S.A.) supplemented with 10% FBS, 100 U/mlL penicillin and 100 μg/ml streptomycin. Cells were passaged every 3 days using 0.25% trypsin.

### RNA interference and transfection

Huh7 and Hep3B cells were transfected with the non-targeting control shRNA (sh-NC) or shRNA targeting LINC00978 (sh-LINC00978) using LipoFit (Hanbio, Shanghai, China) according to the manufacturer’s instructions. Cells were harvested at 36 h post-transfection and RNA interference (RNAi) efficiency assessed by reverse transcription quantitative real-time PCR (RT-qPCR). The shRNA sequences are as follows: sh-NC: 5′-CACCGTTCTCCGAACGTGTCACGTCAAGAGATTACGTGACACGTTCGGAGAATTTTTTG-3′ sh-LINC00978: 5′-CACCGCCCAGATTTAAGGGCTATTTCAAGAGAATAGCCCTTAAATCTGGGCCTTTTTTG-3′.

### RT-qPCR

Total RNA was extracted from human tissues or cultured cells using TRIzol Reagent (Takara, Dalian, China) according to the manufacturer’s protocol. cDNA was synthesized using M-MLV Reverse Transcriptase (Promega, Madison WI, U.S.A.). RNA expression was measured by RT-qPCR using TaqMan Universal PCR Master Mix (Applied Biosystems, Foster, CA, U.S.A.) with the following primers: *GAPDH*, forward: 5′-CGACACTTTATCATGGCTA-3′, reverse: 5′-TTGTTGCCGATCACTGAAT-3′; *LINC00978*, forward: 5′-ACCCTGTGAGCATGATTGGA-3′, reverse: 5′-CTCAAAAGACCCAGATGCCG-3′. Relative quantification was determined by the 2^−ΔΔ*C*_t_^ method using *GAPDH* as the reference gene. All RT-qPCRs were performed in triplicate.

### Proliferation assay

HCC cell proliferation was measured by colony formation and MTT assays. Colony formation assay was performed in triplicate on six-well plates. In brief, transfected HCC cells were re-seeded at 500 per well and allowed to grow for 2 weeks. Afterward, colonies were fixed with 4% paraformaldehyde for 5 min, and stained with 1% Crystal Violet for 10 min at room temperature. For MTT, assays were performed at 24-h intervals on transfected HCC cells seeded at 3 × 10^3^ per well on 96-well plates. For each well, 20 μl of MTT (5 mg/ml, Sigma, CA, U.S.A.) was added and incubated at 37°C for 2 h. The optical density (OD) values were determined at 570 nm with a microplate reader (Tecan Sunrise, Männedorf, Switzerland).

### Flow cytometry

Transfected cells were digested as single cell suspension and fixed with 75% ethanol at 4°C overnight. The fixed cells were stained with propidium iodide (PI) in darkness and treated with RNase A (Sigma, CA, U.S.A.) for 30 min at 37°C. Cell cycle was analyzed by flow cytometry on an FACScan System (BD Biosciences, CA, U.S.A.). For apoptosis, cells were stained with Annexin V-FITC and PI (Sigma, CA, U.S.A.) for 15 min in darkness at room temperature. Cells undergoing early and late apoptosis were quantified on the FACScan System. All flow cytometry experiments were performed in triplicate.

### Human xenograft tumor model

Twenty-four male BALB/c nude mice were obtained from Laboratory Animal Centre of Hebei University and maintained under aseptic barrier conditions. At 6-week-old, Huh7 and Hep3B cells were each transfected with Lenti-shLacZ or Lenti-shLINC00978, and 4 × 10^5^ cells per transfection were subcutaneously injected into the back-skin area of each mouse. Tumors were measured with a vernier caliper every 4 days, and tumor volume was estimated by the formula: volume = 0.5 × (length × width^2^) [28]. Tumor weight was measured after excision from killing mice on a digital scale. The animal protocols were approved by the Committee on Animal Welfare of The Affiliated Hospital of Hebei University.

### Western blot

Total proteins were extracted by complete cell lysis reagent (Keygen Biotech, Jiangsu, China) that supplemented phenylmethanesulfonyl fluoride and PhosSTOP. The protein samples were separated on 10% sodium dodecyl sulfate/polyacrylamide gel electrophoresis gels (SDS/PAGE) and transferred on to 0.22 μm polyvinylidene difluoride membranes (Millipore, MA, U.S.A.). The membranes were incubated with specific antibodies against Bax (Cell Signaling Technology, MA, U.S.A.), Bcl-2 (Cell Signaling Technology, MA, U.S.A.), caspase 3 (Cell Signaling Technology, MA, U.S.A.), p-ERK (Cell Signaling Technology, MA, U.S.A.), ERK (Cell Signaling Technology, MA, U.S.A.), p-p38 (Cell Signaling Technology, MA, U.S.A.), p38 (Cell Signaling Technology, MA, U.S.A.), phospho c-Jun N-terminal kinase (p-JNK) (Cell Signaling Technology, MA, U.S.A.), JNK (Cell Signaling Technology, MA, U.S.A.), GAPDH (Cell Signaling Technology, MA, U.S.A.), and β-actin (Proteintech, U.S.A.), followed by incubation with goat anti-mouse or anti-rabbit HRP-conjugated secondary antibodies (Bioss, Beijing, China). The proteins were visualized by ECL Plus Western Blotting Detection System (Amersham Biosciences, CA, U.S.A.), and band intensity was quantified by ImageJ software.

### Statistical analysis

Statistical analysis was performed on SPSS (SPSS, Inc., Chicago, IL, U.S.A.) or GraphPad Prism 7.0 (GraphPad Software, CA, U.S.A.). Data were presented as mean ± standard deviation (SD) of at least three independent experiments. Student’s *t* test and one-way ANOVA were used for comparing differences between two groups or among three or more groups, respectively. Kaplan–Meier’s method and the log-rank test were performed to compare survival rate. *P*<0.05 was considered to be statistically significant.

## Results

### LINC00978 is up-regulated in HCC tissues and correlates with poor prognosis

We first examined LINC00978 expression in 49 pairs of tumor tissues and adjacent non-cancerous tissues from HCC patients using RT-qPCR. The clinicopathologic data of all patients were presented in Table 1. LINC00978 expression was significantly higher in HCC tumor tissue compared with adjacent normal tissue (Figure 1A). Moreover, LINC00978 expression was significantly higher in HCC patients with advanced clinical stages (Edmondson grading III–IV) than that in HCC patients with early stages (Edmondson grading–II) (Figure 1B). To explore the clinical relevance of LINC00978 expression in HCC, we searched for a correlation between LINC00978 expression and clinicopathological characteristics in HCC patients (Table 1). We set the median LINC00978 expression as a cut-off value and divided 49 HCC patients into LINC00978 high expression group (*n*=26 cases) and low expression group (*n*=23 cases) (Figure 1C).

**Figure 1:** LINC00978 is up-regulated in HCC tissue and it associates with poor HCC overall survival (**A**) LINC00978 expression was up-regulated in 49 cases of HCC tissue compared with adjacent normal tissue, which was measured by RT-qPCR. (**B**) LINC00978 expression was up-regulated in advanced stage HCC patients (Edmondson grading III–IV) than that in early-stage HCC patients (Edmondson grading I–II). (**C**) Relative LINC00978 expression in all HCC tissues. LINC00978 expression level was grouped into low expression (*n*=23 cases) and high expression (*n*=26 cases) using median level as the cut-off value. (**D**) Kaplan–Meier survival curves of HCC patients grouped by LINC00978 expression level. HCC patients with high HCC-tissue LINC00978 expression was associated with lower 5-year overall survival rate.

**Table 1:** Relationship between lncRNA LINC00978 expression and clinicopathological parameters of HCC patients

Parameters	*n*=49	LINC00978 expression		*P*-value
		Low (*n*=23)	High (*n*=26)	
Gender				0.5816
Male	25	10	15	
Female	24	13	11	
Age				0.5521
<50 years	31	14	17	
≥50 years	18	9	9	
AFP (ng/ml)				0.3423*
<400	13	6	7	
≥400	36	17	19	
Tumor size				0.0354*
<5 cm	21	9	12	
≥5 cm	28	14	14	
Histological grade				0.6833
Well	21	10	11	
Poorly/others	28	13	15	
Macro-vascular invasion				0.0565
Yes	17	7	10	
No	32	16	16	
Lymph node metastasis				0.0455*
Yes	33	14	19	
No	16	9	7	
Edmondson grading				0.0243*
I–II	27	12	15	
III–IV	21	11	11	
TNM stage				0.0353*
I–II	17	7	10	
III–IV	32	16	16	

Abbreviations: AFP, α-fetoprotein; TNM, tumor-node-metastasis. *P<0.05 presented as significant difference.

Five-year overall survival was significantly poorer in LINC00978 high expression group than that of low expression group (Figure 1D). In addition, LINC00978 expression was significantly associated with higher tumor size, lymph node metastasis, Edmondson grading, and tumor-node-metastasis (TNM) stage (Table 1). There was no significant association with gender, age, α-fetoprotein level, HCC histological grade, or macrovascular invasion. Taken together, these results showed that LINC00978 was up-regulated in HCC tissue, and high LINC00978 was correlated with poor prognosis for HCC patients.

### LINC00978 is up-regulated in HCC cell lines

We next examined LINC00978 expression in multiple HCC cell lines including SK-Hep1, Bel-7404, Huh7, Hep3B, and HepG2. Consistent with the results in tissue of HCC patient, LINC00978 showed three- to six-fold higher expression in HCC cell lines than that in normal human hepatic cell line LO2 (Figure 2). The results in HCC tissue and HCC cell lines indicated a positive role of LINC00978 in HCC carcinogenesis. Based on the expression profiles, we chose two HCC cell lines Huh7 and Hep3B, which had the highest LINC00978 expression, for subsequent studies.

**Figure 2:** LINC00978 expression is up-regulated in HCC cell lines SK-Hep1, Bel-7404, Huh7, Hep3B, and HepG2 compared with normal hepatic cell line LO2, which was measured by RT-qPCR *P <0.05; **P<0.01 compared with the control group.

### LINC00978 increases HCC cell proliferation

To examine the role of LINC00978 in HCC cells, we transfected Huh7 and Hep3B cells with either non-targeting shRNA (sh-NC) or shRNA against LINC00978 (sh-LINC00978). RT-qPCR showed significant reduction in LINC00978 expression by sh-LINC00978 comparing with sh-NC (Figure 3A,B). We found Huh7 and Hep3B cells that were transfected with sh-LINC00978 showed significantly reduced proliferation capacity than sh-NC, which was measured by the MTT assay (Figure 3C,D) and the colony formation assay (Figure 3E–H). These results suggest that LINC00978 promotes HCC cell proliferation.

**Figure 3:** LINC00978 promotes HCC cell proliferation *in vitro* LINC00978 expression was reduced in HCC cell lines Huh7 (**A**) and Hep3B (**B**) that transfected with shRNA against LINC00978 (sh-LINC00978), comparing with cells transfected with non-targeting sh-NC. LINC00978 knockdown by sh-LINC00978 significantly decreased Huh7 (**C**) and Hep3B (**D**) cell proliferation that was measured by MTT assay. LINC00978 knockdown by sh-LINC00978 significantly reduced colony formation by HCC cell lines Huh7 (**E,G**) and Hep3B (**F,H**). (mean ± SD; *P<0.05, **P<0.01 compared with sh-NC).

### LINC00978 promotes HCC cell cycle progression and inhibits apoptosis

We next examined the role of LINC00978 in regulating HCC cell cycle and apoptosis by flow cytometry. In both Huh7 and Hep3B cells, LINC00978 knockdown induced cell cycle arrest, which was demonstrated by a significant increase in the proportion of cells in G_1_ phase (*P*<0.05) and decrease in proportion of cells in S phase (*P*<0.01) at 48 h after shRNA-transfection (Figure 4A–D). In both Huh7 and Hep3B cells, LINC00978 knockdown significantly increased the percentage of apoptotic cells compared with sh-NC (*P*<0.01, Figure 4E,F). Consistent with the increase in apoptosis by sh-LINC00978, Western blot showed that LINC00978 knockdown significantly increased expression of pro-apoptotic protein Bax, and decreased expression of anti-apoptotic protein Bcl-2 compared with sh-NC (Figure 4G–K).

**Figure 4:** LINC00978 promotes cell cycle progression and inhibits HCC apoptosis (**A**–**D**) LINC00978 knockdown induced HCC cell cycle arrest. Cell cycles of Huh7 (A,C) and Hep3B (B,D) cells transfected with sh-LINC00978 or sh-NC were analyzed by flow cytometry. sh-LINC00978 transfection led to significantly increased proportions of cells at G_1_ phase and decreased proportions in S phase comparing with sh-NC. (**E,F**) Apoptosis in Huh7 (E) and Hep3B (F) HCC cells was significantly increased by LINC00978 knockdown, as determined by flow cytometry. (**G**–**K**) Western blot showing LINC00978 knockdown led to Bax and caspase-3 up-regulation and Bcl2 down-regulation in Huh7 (G,I–K) and Hep3B (H,I–K) cells, normalized to GAPDH (mean ± SD; *P<0.05, **P<0.01 compared with sh-NC).

### LINC00978 promotes HCC tumor growth *in vivo*

In order to test whether LINC00978 regulates HCC carcinogenesis *in vivo*, we compared Lenti-shLacZ and Lenti-shLINC00978-treated HCC tumor growth *in vivo*, using a subcutaneous xenograft tumor model in mice. Huh7 and Hep3B cells that transfected with Lenti-shLacZ or Lenti-shLINC00978 were injected into nude mice subcutaneously, and the volume of xenografts were measured over time. Both of the HCC xenografts developed into visible tumors. We found that the volume of Lenti-shLINC00978-treated HCC xenografts was significantly smaller than that of Lenti-shLacZ-treated tumors (Figure 5). This difference in xenograft growth strongly supports that LINC00978 promotes HCC carcinogenesis *in vivo*.

**Figure 5:** LINC00978 enhances HCC tumor growth *in vivo* (**A,B**) Representative images of subcutaneous HCC tumor xenografts on nude mice at 24 d post-injection of Hep3B (A) and Huh7 (B) cells. (**C,D**) Volume of HCC tumor xenografts in mice injected with Huh7 (C) and Hep3B (D) cells, calculated by length × width^2^ × 0.5. (**E,F**) Weight of HCC tumor xenografts measured after excision from mice (mean ± SD; *P<0.05, **P<0.01 compared with Lenti-shLacZ).

### LINC00978 activates MAPK/ERK signaling pathway in HCC cells

In order to investigate the mechanism between LINC00978 and HCC carcinogenesis, we examined activation of signaling proteins in the MAPK/ERK pathway, which is essential to the proliferation, survival, and differentiation of many cancer types including HCC [29]. We confirmed that LINC00978 is inhibited in Lenti-shLINC00978-treated HCC xenografts than that in Lenti-shLacZ-treated tumors by RT-PCR (Figure 6A). Then the MAPK/ERK signaling pathway was found to be activated (Figure 6B). In both Huh7 and Hep3B cells, LINC00978 knockdown lead to decreased levels of phospho-ERK (p-ERK), phospho-p38 (p-p38) and p-JNK (Figure 6C,D). These data suggest that LINC00978 may partially induce HCC carcinogenesis via activating the MAPK/ERK signaling pathway.

**Figure 6:** LINC00978 activates MAPK/ERK signaling pathway in HCC cells (**A**) LINC00978 is inhibited in Lenti-shLINC00978-treated HCC xenografts than that in Lenti-shLacZ-treated tumors by RT-PCR. (**B**) MAPK/ERK signaling pathway was activated in HCC tissues, compared with peritumor tissues. Protein expression of ERK, p38, JNK, p-ERK, p-p38 and p-JNK were measured by Western blot in Huh7 and HepG2 cells transfected with Lenti-shLINC00978 or Lenti-shLacZ. Lenti-shLINC00978 transfection significantly reduced p-ERK, p-p38, and p-JNK levels in both Huh7 (**C**) and HepG2 (**D**) cells compared with Lenti-shLacZ (mean ± SD; *P<0.05, **P<0.01).

## Discussion

The major result of our study is that lncRNA LINC00978 promotes HCC carcinogenesis. LINC00978 was up-regulated in HCC patient tissues and predicted poor overall HCC survival. LINC00978 promoted HCC cell proliferation and cell cycle progression, inhibited apoptosis *in vitro*, and increased HCC tumor growth *in vivo*. Several signaling molecules in the ERK/MAPK signaling pathway was inhibited by LINC00978 knockdown in HCC cells. Thus, the present data provide strong functional evidence for the regulatory role of a novel lncRNA LINC00978 in HCC pathogenesis.

Given the limited therapeutic choices for HCC, there is an urgent need for developing early diagnostic and prognostic tools. Non-coding RNAs have been recognized as excellent biomarkers for the diagnosis and prognosis of various cancer types including HCC [8,10,30,31]. A previous study found that high LINC00978 expression in breast cancer is associated with poor disease-free survival [25]. Our results suggest the potential use of LINC00978 as an early HCC prognostic marker. However, studies with larger sample sizes are required to further assess its sensitivity and specificity.

A previous study has found that LINC00978 was dysregulated in breast cancer [25]. However, whether LINC00978 dysregulation was causal or simply a marker for tumors was unclear. Fu et al. [24] showed that LINC00978 was a biomarker and an oncogene that promotes gastric cancer progression. Our results are concordant with that conclusion and indicate that LINC00978 is an HCC biomarker as well as a causal factor that extensively involved in promoting a proliferative, pro-survival phenotype essential to HCC carcinogenesis. Notably, the causal role of LINC00978 in tumorigenesis has been reported in other cancer types [23,24,32], suggesting that LINC00978 could have a broad impact on the progression of various cancer types.

The regulatory function of lncRNA depends on lncRNA–DNA, lncRNA–RNA, or lncRNA–protein interactions [33]. However, the target interactors for LINC00978 in HCC are unknown. The murine ortholog of LINC00978, *Morrbid*, was found to regulate the expression of a pro-apoptotic gene *Bcl2l11* in mouse myeloid cells and promote myeloid cell lifespan [27]. While a similar mechanism for LINC00978 in HCC would be concordant with its anti-apoptotic role, i.e., the function of lncRNA is highly cell type-specific and displays vast tissue variation [34]. For example, others found that LINC00978 knockdown inhibited the TGF-β/SMAD pathway in gastric cancer, but we found that LINC00978 knockdown inhibited the MAPK/ERK pathway in HCC cells. Illuminating the exact regulatory target of LINC00978 in HCC will require unbiased transcriptome profiling such as RNA sequencing after RNA depletion of LINC00978, and biochemical studies are necessary to directly capture lncRNA interactions in HCC tissues or cell lines [35].

Recent preclinical data showed that blocking particular signaling molecules in the MAPK/ERK pathway could be beneficial for patients with advanced HCC [36–38], which is regarded as one of the most promising approaches for targeted HCC therapy [39–41]. We found that LINC00978 knockdown inhibited the phosphorylation of several signaling molecules in the MAPK/ERK pathway. Similarly, in colorectal cancer, Ouyang et al. [42] demonstrated that LINC00978 was involved in the P38/MAPK pathway by performing functional annotation based on Gene set enrichment analysis, and they suggested that LINC00978 might promote colorectal cancer cell growth, metastasis, and poor survival via P38/MAPK pathway. ERK, p38, and JNK have been shown to have profound effects on HCC cell differentiation, proliferation, survival, and invasion [40,43–45]. These data suggest that inhibiting LINC00978 could be a desirable therapeutic direction for HCC. However, the mechanisms by which LINC00978 activates MAPK/ERK pathway requires further evaluation.

Our results have a few limitations. First, the HCC tissue was collected from Chinese patients with high prevalence of hepatitis B infection. Given the difference in HCC etiology, whether our findings are applicable to non-Asian HCC patients remains to be verified. Second, our clinical study was based on limited samples, and would have to be validated by larger cohorts with more heterogeneous populations. Third, it is conceivable that LINC00978 may have a wide range of functions in HCC tumorigenesis and may involve additional signaling pathways, which are not identified by the present study.

## Conclusion

Overall, current work identified the role of a novel lncRNA LINC00978 in HCC carcinogenesis. LINC00978 is up-regulated in HCC tissue and it correlates with poor HCC prognosis. LINC00978 promotes the proliferation and survival of HCC *in vitro*, and increases HCC tumor growth *in vivo*, partially by activating the MAPK/ERK pathway.

## Abbreviations

Bcl-2: B-cell lymphoma-2
ERK: extracellular signal-regulated kinase
FBS: fetal bovine serum
HCC: hepatocellular carcinoma
HRP: horseradish peroxidase
JNK: c-Jun N-terminal kinase
LINC: long intergenic non-coding
lncRNA: long non-coding RNA
MAPK: mitogen-activated protein kinase
PI: propidium iodide
RT-qPCR: reverse transcription quantitative real-time PCR
sh-LINC00978: shRNA targeting LINC00978
sh-NC: control shRNA
